# Implementation of Machine Learning Models for the Prevention of Kidney Diseases (CKD) or Their Derivatives

**DOI:** 10.1155/2021/3941978

**Published:** 2021-12-30

**Authors:** Khalid Twarish Alhamazani, Jalawi Alshudukhi, Saud Aljaloud, Solomon Abebaw

**Affiliations:** ^1^University of Ha'il, College of Computer Science and Engineering, Department of Computer Science, Ha'il, Saudi Arabia; ^2^Department of Statistics, Mizan-Tepi University, Tepi, Ethiopia

## Abstract

Chronic kidney disease (CKD) is a global health issue with a high rate of morbidity and mortality and a high rate of disease progression. Because there are no visible symptoms in the early stages of CKD, patients frequently go unnoticed. The early detection of CKD allows patients to receive timely treatment, slowing the disease's progression. Due to its rapid recognition performance and accuracy, machine learning models can effectively assist physicians in achieving this goal. We propose a machine learning methodology for the CKD diagnosis in this paper. This information was completely anonymized. As a reference, the CRISP-DM® model (Cross industry standard process for data mining) was used. The data were processed in its entirety in the cloud on the Azure platform, where the sample data was unbalanced. Then the processes for exploration and analysis were carried out. According to what we have learned, the data were balanced using the SMOTE technique. Four matching algorithms were used after the data balancing was completed successfully. Artificial intelligence (AI) (logistic regression, decision forest, neural network, and jungle of decisions). The decision forest outperformed the other machine learning models with a score of 92%, indicating that the approach used in this study provides a good baseline for solutions in the production.

## 1. Introduction

Chronic kidney disease (CKD) is one of the leading causes of death in recent years, according to a report by the Global Burden of Disease [1]. One in every seven persons has CKD, one of the undiscovered illnesses that have the greatest influence on patients' quality of life and increase the chance of death significantly. The general system of social security in health (SGSSS) has taken chronic kidney disease (CKD) into account [2], as a high-cost pathology for generating a powerful economic impact on the finances of the system, causing a dramatic effect on the quality of life of the patient and their family, including employment repercussions. To reduce the high mortality of CKD, research should be deepened and directed to the initial stages of the disease, analyzing its risk group, with the help of laboratory tests, seeking that patients do not reach the final stages such as dialysis, transplantation, or death [3]. Through automatic learning, the aim is to find a valuable contribution so that an early classification of the disease can be carried out in its initial stages through the results of clinical laboratories, taking advantage of the great potential of automatic learning in the analysis and classification of the data. It is necessary that the technical help tools that are based on data can support the decision-making process in the initial diagnoses quickly, with high precision, and at low cost. With them, the time required for diagnosis is reduced, allowing the patient to receive treatment for the disease before it progresses to a stage of no return.

Machine learning can be broadly divided into supervised learning, unsupervised learning, and reinforcement learning [4]. Supervised learning is the most common form of machine learning used in medical research [5]. Each instance of supervised learning contains an input object (usually a vector) and the desired output value (also known as a supervised signal) [3]. Usually, the algorithms applied for supervised learning are decision trees, naive bayes classification, least squares regression, logistic regression, and vector support machine (SVM) methods (Classifier Sets). Recent studies show that deep neural networks have achieved comparable high performance at the expert level in natural and biomedical image classification tasks [6]. This, coupled with the ability to generate assumptions [7], the adaptability to heterogeneous data set analysis, and open-source deep learning programs that are widely disseminated, makes deep learning play an essential role in promoting medical development [8].

This research work aims to design and implement a machine learning model that, based on data from clinical laboratories, allows predicting the possible diagnosis of CKD in its initial stages, helping reduce the mortality rate and costs for the health system.

## 2. Methodology

In the development of this project, the CRISP-DM® model [9–15] is used, which is the broadest reference guide used in the development of analytical and mining projects to data collected from clinical laboratories. For this, each of the proposed stages will be implemented.

### 2.1. Phase I. Understanding the Business

This phase is divided into four tasks that will help better understand the business, as shown in Figure 1.

#### 2.1.1. Determination of Business Objectives

Chronic kidney disease (CKD) is a type of kidney disease in which there is gradual loss of kidney function over a period of months to years, Initially, there are generally no symptoms; later, symptoms may include leg swelling, feeling tired, vomiting, loss of appetite, and confusion. Complications include an increased risk of heart disease, high blood pressure, bone disease, and anaemia. CKD is associated with a decrease in kidney function related to age and is accelerated in hypertension, diabetes, obesity, and primary kidney disorders. CKD is a global health problem with a high morbidity and mortality rate, and it induces other diseases. As there are no obvious symptoms during the early stages of CKD, patients often do not notice the disease, this being the main feature, eventually leading to a complete loss of kidney function. Early detection of CKD allows patients to receive timely treatment to improve the progression of this disease. As it has been proposed in the objectives of the work, the aim is to develop an automatic learning model for the prediction in the diagnosis of CKD and to contribute to the reduction of significant complications in the disease such as dialysis processes, kidney transplantation, or reaching death. The main criterion of success for this project, with the help of machine learning, is to identify the behaviors or behavior patterns in the initial stages of CKD to improve the quality of life of patients.

#### 2.1.2. Assessment of the Situation

The idea for the approach of this project arises from the current situation regarding the increase in the confirmatory diagnosis of CKD, and lack of treatment or the user's ignorance of its pathologies leads to irreversible kidney failure in the final stages of CKD, such as dialysis for life, financially affecting the health system, as it is a costly treatment that generates the most significant amount of absorption of the resources available for health in Iraq. This could be reduced by using tools such as machine learning to classify ERC from the initial stages. Although the application of machine learning in healthcare and other areas is favorable, the field of kidney disease has not yet exploited its full potential [16–25].

#### 2.1.3. Determination of the Data Mining Objectives

As referenced in the general objective, the technical terms of this project are to design, implement, and deploy a machine learning model that, based on data from clinical laboratories, allows to classify the possibility of a diagnosis of CKD. Through the analysis of laboratory studies that are low-cost for health entities, these data reduce the mortality rate and costs of the health system.

The medical history and the laboratory tests indicate identifying symptoms or signs that can be used as constitutive variables of the problem in CKD patients on a large scale since a large amount of data can be handled without inconvenience. With the initial data, a description and exploration of these are made, verifying that they can be used or have the minimum information to perform the classification, through the analysis of these data and obtain the patients with an incidence of CKD. With the data obtained, a training set is molded. Several tests are carried out that define or determine the most appropriate technique(s) for the classifier and that the results are practical and efficient. With the defined classifier, the predictive models are trained and validated to establish the model with the highest precision for the data, selecting the one that offers the best results. Predictive models often run calculations during ongoing transactions, for example, to assess the risk or opportunity for a particular patient in a way that provides insight into the treatment decision-making.

#### 2.1.4. Production of the Project Plan

The project plan can be found in the schedule annex-project work plan. It describes all the necessary steps, from the problem statement and data collection to its analysis.

### 2.2. Phase II: Study and Understanding of the Data

This section describes the initial data obtained, such as the number of records and fields per record and their identification, each field's meaning, and the initial format's description, as shown in Figure 2.

#### 2.2.1. Collection of Starting Data

The data set used for this project was obtained thanks to the Baghdad Renal Clinic, Iraq, and its manager and legal representative, nephrologist Dr. Ahmad. They allowed and authorized the treatment of these data. The dataset contains 373,770 anonymized samples. In this data set, each sample has 17 variables or predictive characteristics (11 numerical variables and six categorical (nominal) variables).

#### 2.2.2. Explore the Data

To explore the data, a database was created on the Azure platform. The data are imported and connected to the Power BI visualization tool to perform and visualize all the data contained in the data set more harmoniously. Initially, descriptive statistics of the variables that make up the data are carried out. In Table 1, the main characteristics of the variables of the files used are identified; this result was obtained from Python commands within Power BI.

Before starting to process the data set, a set of visualizations is made to help better understand the characteristics of the information being worked with and their correlation. First, the four input characteristics with names “Duration,” “Pages,” “Actions,” and “Value” are displayed in a historical format; it can be seen graphically which values comprise the minimums and maximums and in which intervals the highest density of records is there. As can be seen in the data, the base diseases of CKD are hypertension and diabetes. The data show us that there are many patients with this disease, but hypertension, also known as a silent disease, is highlighted. Considering the obtained results, the highest prevalence of CKD is in women due to their longer life expectancy and reaching the age of risk of CKD (older adult). It is estimated that a quarter of chronic patients present with low hemoglobin in the initial stages of the disease. Epidemiological studies place excess weight as a risk factor for the development of CKD along with other factors. As creatinine rises in your blood average, the percentage of kidney function goes down. For the above reason, it is a significant variable for the diagnosis of kidney disease. As evidenced, the age and weight variables present a high positive correlation, which is not present between hypertension and diabetes mellitus, and no correlation is observed between these variables. There is a low positive correlation for the variables of weight and hypertension, as it also happens between the variables of hypertension with age and diabetes mellitus with age. That is, hypertension and diabetes mellitus are diseases that do not depend on age factor; it can be caused due to family history.

#### 2.2.3. Verification of the Quality of Data

In this section, data verification was performed to determine the consistency of the field values and the amount of distribution of the null values and to find out-of-range values that can generate noise for the process. This verification process was carried out on the entire data set received. In the fields where no records were found, the empty fields were changed to a Null value.

### 2.3. Phase III: Data Analysis and Selection of Characteristics

By having the information from the data, the focus is on identifying the variables to be used. During the data review, a total of 58 variables were found; within these, three variables were identified that were eliminated to preserve the privacy, security, and sensitivity of the patients. Of the 55 remaining variables, those who did not have a sample were eliminated since they would not have any determination if they did not provide information in training. Afterward, a classification was made between the subjective and objective variables. After performing the medical analysis, 38 variables that are not relevant for CKD prediction were eliminated.

With the identification of the scale used to classify patients with CKD, the variables to be used to evaluate a patient according to their degree of severity were determined. The initial list of 58 variables after performing the medical analysis allows us to arrive at a set of 17 variables, which required the expertise of the nephrologist in the elimination process. Within this entire process, these criteria will be used to measure the severity of kidney disease. It is essential to be clear that the judgment of the expert (in this case, the doctor) is crucial to make a final decision about the condition of a patient; for this, the expert will take into account the essential antecedents such as hypertension and diabetes. When the data set is ready, the import is carried out on the experiment that will be carried out in Azure Machine Learning Studio, where the algorithms will be evaluated. Selecting the numeric and non-numeric attributes allows limiting the columns available for a later operation. By having the attributes selected, it is indicated which column will have the values to be categorized or predicted; in the case of this evaluation, the variable stage is used. As indicated in Table 2, it is the one that describes the stage of renal failure in a patient.

Having identified the characteristics of the data set with the most significant predictive power, statistical tests are performed with the Pearson correlation test to determine which columns are more predictive. For this task, the filter-based feature selection module that Azure machine learning brings is used, as seen in Figures 3 and 4, which provides multiple feature selection algorithms, including correlation methods identifying the ordinal and non-ordinal variables.

### 2.4. Phase IV: Modeling

As the next step, the selection process of the machine learning technique that will be used to develop the classifier of patients, this is when the object of this research begins.

According to the effectiveness of the algorithms most used in studies for the diagnosis of diseases, the following algorithms are chosen:

- Logistic regression (LR)
- Artificial neural networks (ANN)
- Forest of decisions (RF)
- Jungle of decisions (DJ)

By having these algorithms, the data set is divided randomly into two parts: training sets and test sets. The experiment is carried out with the split module, (Figure 5) using 70% of the data as training data and 30% is reserved to evaluate the model's efficiency.

Then, the chosen models are trained using the train model tool, an Azure tool used to train a model in a supervised way with the training data set as input to the image model training experiment Figure 6. To these models, the score model is added which is used in Azure for score predictions of a trained model. In each combination of the trained model and the test data, the evaluate model classification model is used to calculate the results confusion matrix Figure 7.

When carrying out this first evaluation of the chosen algorithms, it is verified that the data for the models are unbalanced. For example, in general, precision is the probability that an individual is correctly classified by a test, that is, the sum of the true positives plus the true negatives divided by the total number of individuals evaluated gives acceptable values as observed in Table 3. Still, when verifying the matrices, the values always tend to stage 3.

The SMOTE module is added to carry out the balancing task, a statistical technique that allows increasing the number of cases in a balanced way, taking samples from the characteristic space for each target class and its closest neighbors.

### 2.5. Phase V: Evaluation

The most critical measure of classification algorithms is their accuracy. As observed in the comparative results based on the precision Table 4, it is found that the four classification algorithms were compared. Multiclass logistic regression (LR) achieves the lowest accuracy, 68%, which implies a poor classifier of results.

However, the jungle multiclass decision (DJ) and multiclass neural network (ANN) algorithms work well and show competitive performance with each other.

Although they have reached an accuracy of 75% and 80%, respectively, they fail to show superior performance to the multiclass decision forests (RF) algorithm, which reached an accuracy of 92% that indicates the effective performance in the classification of the ERC dataset used.

## 3. Conclusions

This study explored how a learning model can be used to classify the possibility of a CKD diagnosis.

Consequently, the indirect agreement with the objectives of the project, the CRISP-DM methodology was adapted to the context of the problem so that the different logically organized stages were taken; data collection, pre-processing, learning, evaluation, and selection, which allowed the construction of a model capable of classifying the possibility of a diagnosis of CKD with an accuracy of 93%. As evidenced in the results, the decision forests algorithm has obtained quite optimal results, where predictions of 93% have been obtained. Data preparation is a fundamental step in the process and the absolute precision of the model is directly dependent on this phase. Thanks to the models, we can see how changing the characteristics affects the search for the target value with a simple change of column selection or improvements in the data. The innovation of this work results from the design adjusted to the environment of the health system in Iraq and the pathology of the CKD in our country, with a methodology adapted to the case study and a production architecture proposal for the model with Microsoft Azure tools of form that allows satisfying in the future the scalability of the solution. Furthermore, this methodology could apply to clinical data of other diseases and pathologies inaccurate medical diagnoses. The development of this project allowed the author to acquire more excellent knowledge through both practical and theoretical work about current techniques for the development of machine learning.

This study has limitations, so there is a room for future research. The study did not have a significant data sample due to the restrictions of medical data and its legal effects in Iraq. Continuing with the expansion of the database (increasing the number of examples for each variable) would reduce the limited generalization error for the model and, at the same time, allow the severity of the disease to be detected. This model can be refined with increasing data size and quality. It also opens the space for a variety of studies from other disciplines, such as economic studies around the impact of obtaining a diagnosis in less time to treat the disease in early stages, reducing costs in the health system. In addition, a variety of sociological and clinical studies on the consequences of early CKD management brings about the quality of life of patients and their families. Although the validity of this research is internal, since the document corpus is private and cannot be published for other works, it will help interested professionals with machine learning to carry out their studies in the classification area.

## Figures and Tables

**Figure 1:** Business understanding tasks.

**Figure 2:** Study tasks and understanding of the data.

**Figure 3:** Image data preparation experiment.

**Figure 4:** Modeling.

**Figure 5:** Image data division experiment.

**Figure 6:** Image model training experiment.

**Figure 7:** Evaluation (obtaining results).

**Table 1:** Statistics of the variables.

.	Average	Std.dev	Minimum	25%	50%
Municipality	30328.27	28219.83	5001.00	8001.00	13001.00
Age	73.51	12.01	1.00	67.00	75.00
HTA	1.00	0.00	1.00	1.00	1.00
Albunia	2.50	1.50	0.00	1.00	3.00
Sugar	2.00	1.22	0.00	1.00	2.00
UREA_SANGRE	143.39	86.16	1.00	70.00	139.00
Creatinine	5.78	4.89	0.10	1.70	3.80
Sodium	134.95	20.23	100.00	117.00	135.00
Potassium	4.75	1.30	2.50	3.60	4.80
Hemoglobin	14.40	1.31	12.10	13.40	14.30
DM	0.00	0.00	0.00	0.00	0.00
Weight	77.75	10.00	60.00	70.50	77.20
Stadium	3.14	0.44	3.00	3.00	3.00

**Table 2:** Stadium classification.

Stadium	Description
1	Kidney damage with normal or high filtration
2	Kidney damage with mild decrease in kidney function
3	Kidney damage with a moderate decrease in kidney function
4	Kidney damage with a severe decrease in kidney function
5	Renal failure

**Table 3:** Performance comparison between models.

	Multiclass red neuronal	Decision forest multiclass	Multiclass logistic regression	Multiclass jungle of decisions
General accuracy	0.784	0.831	0.773	0.835
Medium accuracy	0.892	0.887	0.886	0.890
Micro-precision averaged	0.784	0.831	0.773	0.835
Macro-accuracy averaged	0.446	0.691	0.374	0.817
Micro-sensitivity averaged	0.784	0.831	0.773	0.835
Macro-sensitivity averaged	NA	0.617	NA	0.537
Artificial neural networks matrix				
Current class		3	4	5
	3	0.971	0	0.029
	4	0.972	0.001	0.028
	5	0.829	0	0.17
Decision forest matrix				
Current class		3	4	5
	3	0.939	0.033	0.027
	4	0.494	0.417	0.089
	5	0.406	0.1	0.494
			
Logistic regression matrix				
Current class		3	4	5
	3	0.94	0.014	0.046
	4	0.799	0.121	0.08
	5	0.595	0.035	0.37
Jungle matrix of decisions				
Current class		3	4	5
	3	0.987	0	0.013
	4	0.778	0.153	0.069
	5	0.507	0.023	0.471

**Table 4:** Final accuracy and completeness values.

	Accuracy	Completeness
Decision forests	0.922	0.921
Neural networks	0.806	0.800
Logistic regression	0.689	0.689
Decision jungle	0.754	0.750

## Data Availability

The data underlying the results presented in the study are available in the manuscript.
